RETRACTED

# Analyzing the Check-In Behavior of Visitors through Machine Learning Model by Mining Social Network's Big Data

**DOI:** 10.1155/2021/6323357

**Published:** 2021-11-30

**Authors:** Li Hou, Qi Liu, Jamel Nebhen, Mueen Uddin, Mujahid Ullah, Naimat Ullah Khan

**Affiliations:** ^1^School of Information Engineering and Engineering Technology Research Center of Intelligent Microsystems of Anhui Province, Huangshan University, Huangshan 245041, China; ^2^Huangshan Ruixing Automotive Electronics Co., Ltd., Huangshan 245461, China; ^3^School of Communication and Information Engineering, Shanghai University, Shanghai 200444, China; ^4^Prince Sattam bin Abdulaziz University, College of Computer Engineering and Sciences, Al-Kharj 11942, Saudi Arabia; ^5^School of Digital Science, Universiti Brunei Darussalam, Gadong BE1410, Negara, Brunei Darussalam; ^6^Department of Computer Science, Preston University, Islamabad, Pakistan

## Abstract

The current article paper is aimed at assessing and comparing the seasonal check-in behavior of individuals in Shanghai, China, using location-based social network (LBSN) data and a variety of spatiotemporal analytic techniques. The article demonstrates the uses of location-based social network's data by analyzing the trends in check-ins throughout a three-year term for health purpose. We obtained the geolocation data from Sina Weibo, one of the biggest renowned Chinese microblogs (Weibo). The composed data is converted to geographic information system (GIS) type and assessed using temporal statistical analysis and spatial statistical analysis using kernel density estimation (KDE) assessment. We have applied various algorithms and trained machine learning models and finally satisfied with sequential model results because the accuracy we got was leading amongst others. The location cataloguing is accomplished via the use of facts about the characteristics of physical places. The findings demonstrate that visitors' spatial operations are more intense than residents' spatial operations, notably in downtown. However, locals also visited outlying regions, and tourists' temporal behaviors vary significantly while citizens' movements exhibit a more steady stable behavior. These findings may be used in destination management, metro planning, and the creation of digital cities.

## 1. Introduction

The pattern mining and getting meaningful visions from spatial and temporal data has become a vital study subject in subsequent years. Because of the variety of possible uses for location-based social network (LBSN) at the present time, the resultant material has grown significantly quite relevant, particularly from a practical viewpoint. Urban entertainment venues, for example, are linked to revitalizing the inner-city texture and social growth, along with increasing the home-grown economy and liveliness [1, 2]. However, it may face a lot of problems, including the security of social contact between visitors and inhabitants [1]. Excessive entertainment activities can detract from the appeal of various urban places for visitors and inhabitants [3], perhaps exceeding residents' tolerance levels and causing a slew of difficulties [4]. Families around the country voiced similar feelings, accusing visitors for irritations like filth, noise, and congestion in cafés, bars, and public transit [5]. As a result, it is critical to regularly examine visitor actions and behavior to deal with these issues and better prepare for them.

RETRACTED

In the modern era, a large amount of data from every individual's LBSN like WeChat, Twitter, Facebook, and Weibo is available due to the increased usability of smart devices that provide geolocation (longitude and latitude) as well as other demographic information about human behavior such as social media activities, text messages, and phone calls [5]. Researchers have been encouraged to investigate a wide variety of difficulties due to the massive generation of this data to produce genuine models for presenting the spatiotemporal spreading of things. The general residents include people as a source of content due to their engagements and practice of LBSNs by various smart tools that record customers' everyday routines and locations.

We can see behaviors like variations in people's sleep schedules around the entire globe, as well as how citizens from diverse areas of the world spend their winter and summer holidays, and so on, by gathering such data details and examining it per temporal, social, and geospatial elements. In the 1960s, space-based research and urban behavior began to emerge, focusing primarily on the geographically distributed population [6] and geography over time for improvement. They comprehend humans in terms of their behavior, land use, and long-term relationships. Our research encouraged the behavior of urban activities utilizing LBSN data in this examination on the space and behavior of the urban movement. Studies based on daily urban activities in space and time are currently being conducted [7]. Living space, for example, is referred to as a home (the spatial organization of living space and diversity) [8], and a workstation is referred to as a professional. Sports recreation is a leisure space (focuses on the development of time characteristics, recreational area [9], and general entertainment space selection and course of activity) [10, 11]. According to the study mentioned above, the LBSN dataset documents users' everyday lives, activity patterns, and social media usage behaviors and provides geographical and temporal patterns and dynamics connected to regular routines and user behavior.

RETRACTED

The ongoing fast urbanization of the city is also reflected in the LBSN dataset. In one direction, the simple assumption is that people follow a regular daily routine, such as going to work, eating at a favorite restaurant, and returning home via shopping; in recent years, there has been a fast expansion in online social networks (OSNs), resulting in the development of massive amounts of data, allowing us to investigate sectors of big data where data collection and quantity are critical issues. Initially, personal computers were the only way to access social network services (SNSs) [12]. Users can now explore their social networks in limited spaces and while on the move, thanks to improvements in “smart” mobile device technologies. Providing users access to SNSs on sage devices has allowed them to contact us with “friends” whenever, from any location, and with more ease and accessibility [13].

Social media usage has grown in a lockstep with the rising use of cell phones and the Internet, which has expanded people's capacity to move to other places throughout the universe. Social networking platforms usually accept messages, emails, tweets, and many other kinds of communication, encouraging individuals from across the universe to communicate [14]. With the growth of mobile gadget technologies and the extensive usage of smartphones in current history, a substantial revolution in geolocation abilities has happened, pushing consumers to use location-based services (LBSs), culminating in the upswing and adoption of LBSs [15]. Because of the integration of technology fuelled the growth of LBSNs, users of LBSs exchange data about their practices and priorities, as well as “where, what, why, and with whom” they share this information.

OSNs evolved into LBSNs as time passed, and the user needs to be changed, allowing users to communicate their present position (geolocation). One of the first pieces of research on LBSN usage [16] looked into why and how individuals utilize them. Noulas [17] present an empirical analysis of LBSNs, whereas Scellato et al. [18] present an investigation into the spatiotemporal properties of LBSNs. Researchers have been interested in LBSNs because of their capacity to share a user's position and activities. Different forms of study can be done on the data supplied by these services, ranging from giving time-space information to gaining a deeper knowledge of usage trends (the scope of the present research).

RETRACTED

The KDE approach was used to spatially model geolocation data, providing a wider and more versatile paradigm for density assessment [19]. The KDE technique is well known for evaluating spatial point patterns. In many cases, KDE with spatially adjustable bandwidths is preferred to KDE with invariant bandwidths. However, establishing adaptive KDE bandwidth is highly computationally expensive, especially for large-sample point pattern analysis. We used density estimation maps to demonstrate the influence of multivariate density (KDE) in this work. We mined Weibo data with KDE to illustrate users' check-in patterns. We examined several components of LBSN data to determine the check-in frequency for season-based entertainment venues and investigate density in Shanghai over a given period.

Using LBSN data, we examined check-in behavior in 10 Shanghai districts: Changning, Baoshan, Jingan, Huangpu, Hongkou, Putuo, Yangpu, Minhang, Xuhui, and Pudong New Area. The main reason for choosing these ten districts is because these are all connected to the Shanghai city center. We used a dataset from Weibo for our real investigation, one of China's most important social media networks. Amongst our contributions, the check-in density of visitors for a trial of the common residents of Shanghai and temporal behaviors for regularly oriented rate and gender gaps. This research might help in various fields, such as urban functions, amusement studies, urban sustainability, growth, and backup response, which depend on crowd densities in the metropolitan and upcoming work in these regions.

### 1.1. Study Area and Dataset

Shanghai, China (placed between 30°40′-31°53′ N and 120°52′-122°12′ E [37, 46]) is on the Yangtze River Delta's eastern border [20–22]. Shanghai has a total size of 8359 km^2^, and its gross domestic product (GDP) in 2018 was 480 billion dollars (USD). The research area is shown in Figure 1.

Shanghai was divided into 16 districts in 2016: A state (Chongming) and 15 districts (Fengxian, Minhang, Huangpu, Jingan, Putuo, Hongkou, Jinshan, Changning, Jiading, Songjiang, Qingpu, Baoshan, Yangpu, Xuhui and Pudong New Area) [23]. This study considers Shanghai's ten linked districts (Baoshan, Xuhui, Changning, Huangpu, Minhang, Jing'an, Yangpu, Putuo, Hongkou, and Pudong New Area). Changning, Huangpu, Putuo, Hongkou, Xuhui, Jing'an, and Yangpu are all located in Puxi (Huangpu West). These seven regions are collectively considered as Shanghai's city centre. The study's data originated from the Chinese microblog “Weibo.” This location-based network places a premium on coordinating the user's present position with geospatial bring together, which are real-world coordinates supplied by the client. Users joined the program by signing in, just as they would in any other LBSNs, and chatting on the network. Weibo is one of China's top popular LBSNs, had an exponential surge in activity and recognition immediately after its launch on August 14, 2009, and has since got matured. We picked those Weibo records that were not only China's largest LBSN but also have vast geodata of many techniques and provide multiple social features that entice users to check in regularly. Weibo reported that over 500 million recorded users used the site regularly in 2018, with 462 million daily users in December of 2018. The most current authorized estimate of the figure of everyday active subscribers was 1 trillion in 2018.

RETRACTED

As a result, we must focus on users who use the program regularly to investigate user activity patterns. The data gathered through the use of LBSN applications raises serious privacy fears and imposes significant strict limitations. In China, it is extremely difficult to find open and trustworthy geolocation-based data. The LBSN dataset for this paper was obtained from Weibo between July 2014 and June 2017. Weibo offers an empty geodatabase that can be accessed via the Weibo API, written in Python [24].

Because Weibo has a public geodatabase, the dataset includes user IDs, dates, times, geolocations (longitude and latitude), classifications, and locales. As a consequence of the clients' confidentiality, no confidential information is available. Check-in data tracks users' daily movement patterns and behaviors, reflecting the average person's everyday living activities [25]. Shanghai was considered as the research location because it has a high frequency of check-ins and involved customers. From July 2014 to June 2017, 138,228 check-ins were gathered inside the administrative borders of Shanghai using the application programming interface (API). Weibo data was extracted to remove noise, impersonated users, and incorrect entries. To address the issue of uniqueness and the relevance of the dataset, the following parameters were used for data preparation and cleaning:

- The geographical position of data be located in only in Shanghai
- Each record requirement has a user ID and geolocation (latitude and longitude)

Given the heterogeneity problem, it is critical to limit the sample of users to active people to attain a greater level of predictive value.  Table 1 displays the user ID, latitude, and longitude from the dataset used in our research.

## 2. Methodology

### 2.1. Data Acquisition and Preparation

The vital objective of the data gathering and storage stage was to gain a massive quantity of facts. Using a Python-based application programming interface (API), the data gathered in the data collection activity was transmitted in various JavaScript Object Notation (JSON) file layouts.  Figure 2 depicts the data collecting process flow.

RETRACTED

JSON is a small data interchange format that sends data objects using human-readable language, whereas Java is an object-oriented programming environment [26]. The data was transformed into a single file in CSV (comma-separated values) style for further processing and analysis using the specified software. All of the participants' details, including geolocations, could be listed saved in the database. We gathered the data in CSV style and then used a criterion for the relevance of the results.  Figure 3 depicts the criterion figure.

## 3. Sequential Model

After transformation of data and performing all preprocessing steps, we researched and also applied different models which lead us to the experience of selecting an optimal model for getting maximum accuracy and minimum loss. First of all, we have applied a famous decision tree model of which we got 62 percent accuracy. The limitation there was we were unable to find the loss. The confusion matrix for the decision tree shown true positive is equal to 682, true negative is equal to 8404, false positive 419, and false negative 254. Secondly, we have searched for another model and come to the conclusion to select naïve Bayes classifier of which we got accuracy of 49 percent which was not expected. The confusion metrics where we have true positive is equal to 2990, true negative is equal to 3940, false positive is equal to 3081, and false negative is equal to 2380. Thirdly, a random forest model was selected for training the model of which we have gotten similar accuracy like decision tree. Finally, we transformed our focus to tensor flow and there we selected the sequential model dividing data into training, testing, and validation chunks. We successfully achieved the maximum accuracy 90.18% with 25 number of epochs. This accuracy is significant and satisfying in contrast to other models. It can be seen in Figure 4.

Sequential model loss function was calculated with 25 epochs' loss of 13.61% which has been noticed. During training, initial loss was above 70% and accuracy was 48.44%. After tuning, loss falls to a minimum level given above and accuracy reached to optimum position of 90.18%.  Figure 5 depicts the results.

### 3.1. Social Media Data Analytics Framework

Figure 6 depicts our wide spatiotemporal analysis paradigm. The first component is divided into two parts: data collecting (downloading data from Weibo) and data filtering. The LBSN data will next be examined.

RETRACTED

Following that, the spatial distribution characteristics of these locations were examined using the ArcGIS 10.6.1 software. The study used ArcGIS 10.6.1 software (Environmental Systems Research Institute, Inc., Redlands, CA, USA) and a map of Shanghai generated in 2016 as a working base map with the Geodetic Coordinate System WGS1984.

### 3.2. Analytical Method

#### 3.2.1. Kernel Density Estimation

KDE is a nonparametric technique for calculating intensity from an arbitrary illustration of data. KDE computes even circulations by eliminating local noise to a certain extent, decreasing inaccuracy by giving a nonparametric possibility allocation with optimal frequency. KDE is a density estimate approach that has been broadly explored for the study of many elements of location-based social media data such as establishing city borders, user movement and movement designs, point of interest suggestion, and check-in habits. For modeling spatial densities, the KDE method has also been used in fields such as health, marketing, and environment [19, 21, 27]. KDE has been used in analyzing the patterns of visitors in green parks [25, 28–32].

Let *E* be a set of historical data where *e*^*j*^ = <*x*, *y*> is the geocoordinate of a location, 1 ≤ *j* ≤ *n* for an individual *i*. *h*_*j*_ is the Euclidean distance to *k*-th nearest neighbor *e*^*j*^ in the training data. The KDE is expressed as follows;

(1) $$\begin{array}{c} f_{\text{KD}}\left(e\;|\;E\right)=\frac{1}{n}\overset{n}{\underset{j=1}{\sum }}K_{h^{j}}\left(e,e^{j}\right), \end{array}$$

(2) $$\begin{array}{c} K_{h}=\frac{1}{2\pi h}\exp\left(-\frac{1}{2}{\left(e,e^{i}\right)}^{t}\overset{-1}{\underset{h}{\sum }}\left(e,e^{i}\right)\right). \end{array}$$

## 4. Results

With residents of 22,125,000 people and a land area of 4,015 square kilometers, Shanghai City is one of the world's fastest rising cities [9, 33]. It has compiled the entertainment check-ins data over three years. Every check-in was allocated to the class that best matched the entertainment and amusement activities carried at that location, such as movie, KTV entertainment hall, theatre, and Disney Park.  Figure 7 depicts the total number of check-ins.  Figure 7(a) displays the entire quantity of check-ins, and it can be observed that a few check-ins are not included in our research region. Still, we cleaned the data according to our research region, and all check-ins conducted outside Shanghai's ten districts have been deleted.

We use KDE to study the spatial variation of check-in data and ArcGIS to visualize the Weibo geolocation check-in dataset.  Figure 8 depicts the total check-in intensity in Shanghai from July 2014 to June 2017. Sections coloured in black signify a larger quantity of people, a higher frequency of action, and a greater awareness of social media use. It is no surprise that the seven districts of Shanghai's city center appear denser than the other three districts, although the area of the three districts is larger.

RETRACTED

Figure 9 depicts temporal variations in the number of visits over the course of 24 hours. Although visitors contributed at all times of day, the largest number of check-ins was reported 12 A.M., as well as between 8 P.M. and 11 P.M. among the amusement places studied.

Figure 10(a) depicts the amount of check-ins for each day, and it can be observed that weekends have a larger quantity of check-ins than weekdays.  Figure 10(b) depicts the everyday number of check-ins based on seasons, and it can be seen that there is a higher number of check-ins on weekends in spring.

Check-ins are distrusted at the district level for a more precise picture of amusement place dispersal in Shanghai City.  Figure 11 displays that the distribution of check-ins is maximum in the region of Pudong, followed by the district of Huangpu. The explanation for this tendency is because the Pudong new area district is greater in size than the other districts. Another thing to keep in mind is that the distribution of check-in is higher in the downtown area than in the suburbs.

Figure 12 depicts the total check-ins made every month. It can be witnessed that the months of April, May, and June have a higher number of check-ins than the other months. The check-ins in the months of November, December, and January are lower because of cold weather.

According to comparable research, substantial seasonal changes in user check-ins have been discovered, and many factors have been investigated in an attempt to explain these patterns [34–37].  Figure 13(a) indicates that an advanced amount of check-ins was made at entertainment venues all over the summer and spring. It is important noticing that check-ins are somewhat fewer in the winter than they are in the autumn.  Figure 13(b) depicts the gender differences in seasons, demonstrating that females are more energetic than males in all seasons.

## 5. Discussion

Weibo data, per the findings, is a great resource for assessing the quality of urban amusement and researching spatiotemporal aspects. The advantage of employing social media records for amusement check-in research is that we may obtain qualitative and large-scale statistics of the whole town.

This research used geotagged social media check-in data as a proxy to estimate the number of entertainment venue trips in Shanghai as a case study. This method is less time-consuming and labor-intensive than time-consuming and labor-intensive assessments, and it can provide an exceptional geographical range. We were not capable of defining whether there is a positive link between check-in data and visits seen in urban scheduling and assessment since we lacked accessibility to actual tourist figures.

RETRACTED

It is a big problem since, unlike old-style register data, social media data does not typically provide direct facts such as race and marital status; nevertheless, methods exist to extract them indirectly. The link between the amount of Weibo check-ins and actual visits may vary amongst entertainment venues.

Due to privacy and personal security concerns, the availability of data is a key barrier for LBSN research. The possibility for LBSNs to disclose users' and their friends' current geolocation poses major privacy issues. Individuals are concerned about privacy, but so are organizational or corporate users that exchange content through LBSNs. Private information is sometimes provided freely or unwittingly. Although data is periodically collected by providing unique privileges and benefits to customers in return for their details, it is never often true. The position of a user can be discovered via LBSN services, for example, WeChat Nearby.

To the best of our understanding, this is the first case study that examines the utilization of amusement facility visits in terms of check-in activity for a substantial number of locations in Shanghai using Weibo data. The wide geographical area of the study provides vital information that may help planning and development in other large cities by providing more entertainment venues where people wish to visit.

## 6. Conclusion

We examined the dispersion of users' check-ins in ten distinct districts of Shanghai, emphasizing various elements of georeferenced data. The research region and amusement site check-in datasets were subjected to kernel density estimation. According to our findings, people prefer to attend the entertainment venues in Shanghai's city center, divided into seven districts. The months of April, May, and June have more check-ins comparing with other months. Visitors mostly like to visit in spring and summer, and female visitors are more active. Pudong new area and Huangpu are denser districts than others, and weekends have more check-ins than other days. To conclude, it has been found that sequential model was relatively optimum for training on the data we have used in this research. Using sequential model, we achieved accuracy of 90%. The study may be useful in identifying more congested locations in Shanghai so that controlling or management establishments can observe and assist such regions more effectively, particularly in events, community actions, urban development, and so on.

RETRACTED

Numerous features can be investigated additional in the coming era; the study could be conducted in different characteristics like gender, site classifications, and spatial distribution multiple times with further reasons comprising age, earnings, marital status, etc. It could also highlight the focus elements in the research region to assess the spatial distribution of consumers.

## Figures and Tables

**Figure 1:** Study area.

**Figure 2:** Data acquisition.

**Figure 3:** Criteria.

**Figure 4:** Accuracy of sequential model.

**Figure 5:** Loss function of sequential model.

**Figure 6:** Methodology.

**Figure 7:** (a) Total check-in. (b) Filtered check-in.

**Figure 8:** Check-in density.

**Figure 9:** Hourly check-in.

**Figure 10:** (a) Daily check-in. (b) Daily check-in in seasons.

**Figure 11:** Check-ins' distribution in districts.

**Figure 12:** Seasonal variations were studied for the months of fall, winter, spring, and summer.

**Figure 13:** (a) Number of check-ins during seasons. (b) Gender difference.

**Table 1:** The example of features in the dataset.

User ID	Activity	Date	District	Lon	Lat	Gender	Time	Day
1.78*E* + 09	Amusement	5/8/2017	Xuhui	121.4487	31.19813	M	2 : 20 : 12	Mon
3.06*E* + 09	Amusement	6/8/2016	Yangpu	121.5208	31.29679	F	18 : 20 : 23	Thu
2.46*E* + 09	Amusement	12/5/2015	Huangpu	121.4634	31.21838	M	7 : 25 : 40	Wed
1.78*E* + 09	Amusement	8/24/2014	Pudong	121.5592	31.24204	M	3 : 30 : 45	Mon

## Data Availability

The Weibo check-ins data used to support the findings of this study are available from the corresponding author upon request.
